# Swin-YOLOv5: Research and Application of Fire and Smoke Detection Algorithm Based on YOLOv5

This article has been retracted.

**DOI:** 10.1155/2022/6081680

**Published:** 2022-06-24

**Authors:** Shangjie Ge Zhang, Fengxi Zhang, Yuyang Ding, Yu Li

**Affiliations:** ^1^College of Science, Northeast Forestry University, Harbin 150040, China; ^2^College of Telecommunications Engineering, Xidian University, Xi'an 710126, China; ^3^College of Foreign Languages, Northeast Forestry University, Harbin 150040, China

## Abstract

Accurate monitoring of fire and smoke plays an irreplaceable role in preventing fires and safeguarding the safety of citizens' lives and property. The network structure of YOLOv5 is simple, but using convolution to extract features will lead to some problems such as limited receptive field, poor feature extraction ability, and insufficient feature integration. In view of the current defects of YOLOv5 target detection algorithm, a new algorithm model named Swin-YOLOv5 was proposed in this work. Swin transformation mechanism was introduced into YOLOv5 network, which enhanced the receptive field and feature extraction ability of the model without changing the depth of the model. In order to enrich the feature map splicing method of weighted Concat and enhance the feature fusion ability of model pairs, the feature splicing method of three output heads of feature fusion layer network was improved. The feature fusion module was further modified, and the weighted feature splicing method was introduced to improve the network feature fusion ability. Experiments showed that, compared with the original algorithm, the rising rate of mAP@0.5 (mean average precision, IoU=0.5) of the improved algorithm was 0.7%, the mAP@0.5:0.95 was increased by 4.5%, and the target detection speed with high accuracy was accelerated by 1.8 FPS (frames per second) under the same experimental dataset. The improved algorithm could more accurately detect the targets that were not detected or detected inaccurately by the original algorithm, which embodied the adaptability of real scene detection and had practical significance. This work provided an opportunity for the application of fire-smoke detection in forest and indoor scenes and also developed a feasible idea for feature extraction and fusion of YOLOv5.

## 1. Introduction

As one of the most frequent and widespread major disasters threatening public safety and social development, fire caused serious casualties and property losses [1, 2]. In 2021, for example, there were 748,000 fires in China, with 1,987 deaths and 2,225 injuries, and the direct property losses amounted to 6.75 billion Chinese Yuan [3]. In order to avoid causing more casualties, it is substantial to detect and douse the fire at the early stage. For the past few decades, the research on fire detection has made rapid progress, such as lidar detection of smoke [4, 5] and analysis and detection of fire gas [6, 7]. With the frequent development of target detection and the continuous improvement of computer computing power, researchers have gradually shifted from traditional sensor detection to deep learning target detection. Chung and Le [8] employed a “false color” technique to detect large-scale pollution incidents through satellite images. Li et al. [9] developed forest fire-smoke recognition based on satellite remote sensing technology by studying artificial neural network and multi-threshold technology. Treyin et al. [10] used the boundary modeling in wavelet domain to detect the flame in infrared (IR) video, which reduced the false alarm caused by ordinary bright moving objects. Muhammad et al. [11] proposed a CNN classification network model for detecting whether there is a flame, but the video images obtained in actual use contain a large number of backgrounds, which interfered with the feature extraction of the classification network, and the accuracy of the model was low.

Among convolutional neural networks (CNNs), YOLO network [12] is widely applied in various fields because of its fast detection speed and high accuracy and is also gradually used in fire detection [13, 14]. Cai et al. [15] refined the residual module with efficient channel attention module, added DropBlock after each convolution layer, and finally proposed a smoke model with strong robustness and high accuracy. At present, there are few cases of YOLOv5 used for fire-smoke detection.

The difference between four versions of YOLOv5 (v5s, v5m, v5l, and v5x) lies in the depth and width settings of the model. For YOLOv5s and YOLOv5m, there are relatively few convolution layers, and the output of feature layer cannot extract the target features well. For YOLOv5l and YOLOv5x, although the deeper semantic features can be extracted by stacking more convolutions, the model detection speed can be improved, and the stacking convolution layers will increase the complexity of the model, thus reducing the speed of model detection.

In this study, the Swin transformer mechanism [16] was introduced, which enhanced the receptive field of the model without changing the depth of the model and could extract target features more accurately and fluently. In addition, we modified the feature splicing method of three output headers of the feature fusion layer network and employed the feature graph splicing method with weight Concat to further enhance the feature capability of the model pair. In the output part of the three detection headers of the network, in order to make better use of the global feature information, this study applied Swin transformer to the three detection headers of the network to further improve the mAP of the model. The improved model has developed a convenient idea for feature extraction and fusion of YOLOv5. The further research direction is to optimize the model structure (including replacing the network model), combine infrared dual-band image monitoring [17, 18], Internet of Things transmission, and the improved automatic fire monitor, manufacture supporting hardware equipment, intelligently detect the initial fire, automatically extinguish the fire and give an alarm, and conduct the simulation experiments, which really provides a possible opportunity for the application of Swin-YOLOv5 model or its optimized substitute in fire-smoke detection in scenes including forest and indoor.

The improved model provides a convenient and feasible idea for feature extraction and fusion of YOLOv5, which is of great significance for fire-smoke detection. The next step is to continuously improve the network and hardware design in combination with relevant topics, so as to provide possible opportunities for the application of Swin-YOLOv5 model or its optimized alternatives in many scenarios such as forest and indoor smoke detection.

## 2. Principle and Experiment

### 2.1. Principle of YOLOv5

Unlike YOLOv3 [19] and YOLOv4 [20], the ground truth of YOLOv5 can be predicted across layers. If there are multiple prediction frames in a certain target, the non-maximum suppression (NMS) algorithm [21] is used to remove the prediction frames with high overlap and low score. As shown in Figure 1, YOLOv5 has a simple network structure, mainly including backbone and head, in which the backbone is used to extract the features of the input picture, and the head is used to further fuse the features extracted by the backbone to obtain richer target features, so as to realize the prediction of the target.

YOLOv5 is a target detection algorithm based on anchor [22]. In order to constrain the center point of the bounding box in the current grid, the sigmoid function is used to process the offset value, which can be ensured to be between 0 and 1. The specific calculation formula is as follows:

(1) $$\begin{array}{c} b_{x}=2\sigma \left(t_{x}\right)-0.5+c_{x},\\ b_{y}=2\sigma \left(t_{y}\right)-0.5+c_{y},\\ b_{w}=p_{w}{\left(2\sigma \left(t_{w}\right)\right)}^{2},\\ b_{h}=p_{h}{\left(2\sigma \left(t_{h}\right)\right)}^{2}, \end{array}$$

where *p*_*w*_, *p*_*h*_ denote the width and height of the anchor (the initial value of the target width and height) and *b*_*w*_, *b*_*h*_ are the true width and height of the target. The parameters of the relative width and height of the output network are indicated by *t*_*w*_, *t*_*h*_, and *t*_*x*_, *t*_*y*_ represent the offset values of the target center point of the network output relative to the grid. *c*_*x*_, *c*_*y*_ are the letters representing the coordinates of the upper left corner of the current grid, and *b*_*x*_, *b*_*y*_ symbolize the coordinates of the real center point of the target, respectively.

### 2.2. Experiment

This work reveals an improved YOLOv5 target detection algorithm (Figure 2) which can be used for fire-smoke detection, mainly including the following three points:

① The Swin transformer mechanism was introduced to enhance the receptive field and the feature extraction ability of the model without changing the depth of the model.
② The feature splicing method of the output heads of the feature fusion layer network is modified, which enriches the feature graph splicing method with weight Concat and enhances the feature fusion ability.
③ The Swin transformer was used in the three detection headers of the network, and the global features of the features were fully integrated before the output of the network to improve the mAP of the model.

#### 2.2.1. Swin Transformer

Some studies have shown that convolution operation merely extracts features from local neighborhood but omits global feature information [23–25]. For the target detection task, it is necessary to build a larger-scale dependency model by stacking multiple convolution layers, so as to gather all local features extracted by convolution to obtain deep semantic features. On the one hand, the method of stacking multiple convolution layers can effectively improve the ability of the network to extract target features, but on the other hand, it will lead to the deepening of the network layer and the increase of computation.

In NLP (natural language processing), the self-attention mechanism [26] can extract context information of text and learn richer semantic features, so introducing self-attention mechanism into computer vision can be considered. For the self-attention mechanism of a single header, the output of each pixel *y*_*ij*_ ∈ *R*^*d*_*out*_^ can be calculated by the following formula:

(2) $$\begin{array}{c} y_{ij}=\sum_{a,b\in N_{k}\left(i,j\right)}{\text{softmax}}_{ab}\left(q_{ij}^{T}k_{ab}\right)v_{ab}, \end{array}$$

where *q*_*ij*_=*W*_*Q*_*x*_*ij*_, *k*_*ab*_=*W*_*K*_*x*_*ab*_, *v*_*ab*_=*W*_*V*_*x*_*ab*_ implied linear changes of pixel points *ij* and surrounding pixels and *W*_*Q*_, *W*_*K*_, *W*_*V*_ ∈ *R*^*d*_*out*_×*d*_*in*_^ are network parameters that the network needs to learn.  Figure 3 presents a schematic diagram of multi-head self-attention mechanism.

Compared with NLP, the scale of computer vision has a wide range, requiring greater resolution, and the computational complexity of transformer in computer vision field is tedious [16]. The self-attention mechanism of the transformer can effectively capture global features. The Swin transformer constructs a hierarchical feature map, which introduces the transformer into computer vision without more computation, and the image size has linear computational complexity.

As shown in Figure 4(a), Swin transformer constructs a hierarchical representation by gradually merging adjacent patches in a deeper transformer layer starting with small patches (gray outline). The Swin transformer model can make intensive prediction conveniently by using hierarchical feature maps. The linear computational complexity is realized by locally calculating self-attention (red outline) in the non-overlapping window of the image partition, rather than on all patches of the whole image. The number of patches in each window is fixed, so the complexity is linearly related to the image size. One of the key design elements of Swin transformer is its shift of window partition between successive self-attention layers, as shown in Figure 4(b). The shift window bridges the window of the previous layer, provides the connection between them, and significantly enhances the modeling ability.

Based on the above factors, the work in this paper introduced Swin transformer as one of the layers into YOLOv5 network structure (Figure 2). The third layer in the backbone was replaced by SWinTR, which was used to increase the receptive field of the network and enable the backbone to extract more global and richer features. In the feature fusion part, the original C3 network structure was replaced by SWinTR at the three output detection headers of the network, which could obtain the global semantic information of the feature map.

#### 2.2.2. Weight Concat

In the deep learning network, the fusion of different scale feature layers is an effective strategy to realize the feature complementarity between feature layers. Lower-level features show higher resolution but lower semantics and more noise. High-level features that have been convolved many times display stronger semantic information, but because of the low resolution of feature map, the perception ability of details is dissatisfactory. The feature fusion of each feature layer can enrich the image features, enhance the feature representation ability of the feature layer, and improve the performance of the target detector [27, 28]. In YOLOv5 model, different feature maps are spliced by simple feature maps stacked by Concat, which affects the feature fusion effect of the network, and the model cannot select more effective feature maps for output. Therefore, this work proposed a weighted feature map splicing method WConcat:

(3) $$\begin{array}{c} \text{output}=\text{conv}\left(\delta \left(\overset{1}{\underset{i=0}{\text{cat}}}\left(w_{i}x_{i}\right)\right)\right),\\ w_{i}=\frac{w_{i}}{\left(\sum_{j=0}^{1}w_{j}+\xi \right)}. \end{array}$$

Figure 5 shows the mosaic mode diagram of WConcat. The feature maps x1 and x2 are spliced after W weight, respectively, then non-linearized by relu activation function, and finally adjusted by a 1^*∗*^1 convolution to get the output. This method can make the network fully integrate the features of different feature maps, and the grid has stronger feature expression ability.

## 3. Results and Discussion

The hardware environment and main software configurations used in this work are shown in Table 1, and the hyperparameter settings used in the experiment are shown in Table 2.

We use AP as the evaluation index of each defect category and map@0.5 as the measurement index of the whole model:

(4) $$\begin{array}{c} P=\frac{\text{TP}}{\left(\text{TP}+\text{FP}\right)},\\ R=\frac{\text{TP}}{\left(\text{TP}+\text{FN}\right)}. \end{array}$$

The curve with P (precision) as the ordinate and *R* (recall) as the abscissa is the P-R curve, which is one of the important indexes for evaluating the performance of the model. The AP value can be obtained by PR curve:

(5) $$\begin{array}{c} AP=\int_{0}^{1}p\left(r\right)dr. \end{array}$$

Accordingly, the measurement index of surface defect target detection can be obtained according to the following formula:

(6) $$\begin{array}{c} \text{m}\mathrm{AP}=\frac{1}{n_{j}\sum_{j=1}^{n_{j}}AP_{j}}. \end{array}$$

The algorithm proposed in this work is trained and verified by using the fire-smoke dataset, which comes from the open source network. The dataset contains 16,503 training pictures, of which 14,715 are used for training and 1,788 are used for verification. The distribution of each category in training dataset and verification dataset is shown in Table 3.

We use the experimental environment shown in Table 1 and the hyperparameters described in Table 2 and use the dataset partition method in Table 3 to train YOLOv5 before and after improvement, respectively. The training results are shown in Figure 6.

Table 4 shows AP value and mAP value more intuitively, which is based on Figure 6. Compared with the original model, the improved model has some advantages. mAP@0.5 of the improved model is 0.7% higher than before, mAP@0.5 : 0.95 is 4.5% higher, and the FPS is 1.8 higher. According to Figure 7, it can be analyzed that under the same experimental dataset, the model modified by Swin-YOLOv5 algorithm can detect the target more accurately, which is not detected or inaccurate by the original model.  Figure 7(a) of the detection results of the original YOLOv5 model shows a rather low detection accuracy (they are all lower than 60%), and the smoke in the picture below cannot be detected, while Figure 7(b) detected by the modified YOLOv5 model shows a relatively high detection accuracy, and the smoke in the picture below can be detected obviously. Considering the requirements of the real environment, compared with the original model, the application ability of the modified Swin-YOLOv5 model in the scenes that need to detect smoke and fire is more worthy of recognition.

## 4. Conclusions

In this paper, an improved algorithm Swin-YOLOv5 based on YOLOv5 was proposed to detect fire and smoke in conflagration accident. Swin transformer feature extraction layer was introduced to enhance the feature extraction ability of the model. A new feature map fusion mechanism was imported to enhance the fusion ability of features and make full use of the features extracted by backbone to realize target detection. For the feature fusion layer, Swin transformer was used to fuse the global information of the summarized feature and improve the mAP of the model. Experimental results showed that mAP@0.5 of target detection model improved by Swin-YOLOv5 algorithm proposed in this paper was 0.7% higher than that of the original algorithm, mAP@0.5 : 0.95 was 4.5% higher, and the high-precision target detection speed was 1.8 FPS higher. In addition, the improved model had better performance than the original model, which was manifested in more accurate detection and more detected objects. The improved model develops a convenient and feasible idea for feature extraction and fusion of YOLOv5, which is of great significance for fire-smoke detection. The further work is to continue to improve the network and design the hardware in combination with related topics, so as to provide possible opportunities for the application of Swin-YOLOv5 model or its optimized substitutes in many scenes such as forest and indoor smoke detection.

## Figures and Tables

**Figure 1:** Structure diagram and prediction structure coding diagram of YOLOv5.

**Figure 2:** The target detection algorithm of improved YOLOv5.

**Figure 3:** The schematic diagram of multi-head self-attention mechanism.

**Figure 4:** Hierarchical representation (a) and sliding window (b) of Swin transformer.

**Figure 5:** Splicing mode diagram of the WConcat.

**Figure 6:** Comparison of results before (a) and after (b) the improvement of YOLOv5.

**Figure 7:** The results of the original ground truth bound (a) and the network detection candidate bound (b).

**Table 1:** Hardware and software configuration of experimental environment.

Name	Parameter
GPU	Tesla V100 32G
CPU	Intel(R) Core(TM) i9 CPU @ 2.30 GHz
OS	Linux Ubuntu 16.04
Deep learning framework	PyTorch 1.7.1+cuda101
Programming language	Python 3.7

**Table 2:** Experimental hyperparameter configuration.

Parameter	Value
Learning rate	0.001
Momentum	0.93
Weight attenuation	0.0005
Iterations	100
Batch size	20
Picture size	640 *∗* 640
Learning rate decay strategy	Cosine

**Table 3:** Label distribution of dataset.

Category	Smoke	Fire
Training set label distribution	10800	3915
Verification set label distribution	1189	599

**Table 4:** Data of experimental results.

	Smoke (AP)	Fire (AP)	mAP@0.5	mAP@0.5 : 0.95
Before	0.780	0.673	0.727	0.382
After	0.797	0.672	0.734 (+0.7%)	0.427 (+4.5%)

## Data Availability

The raw data supporting the conclusions of this article will be made available by the authors, without undue reservation.

## References

[1] Lundquist P., Rammer L., Sörbo B. (1989). The role of hydrogen cyanide and carbon monoxide in fire casualties: a prospective study. *Forensic Science International*.

[2] Lasanta T., Cerdà A. (2005). Long-term erosional responses after fire in the Central Spanish Pyrenees. *Catena*.

[3] Fire and Rescue Department Ministry of Emergency Management[Eb/Ol] (2022). Fire and Rescue Department Ministry of Emergency Management[Eb/Ol]. https://www.119.gov.cn/article/46TiYamnnrs.

[4] Utkin A. B., Fernandes A., Simões F., Lavrov A., Vilar R. (2003). Feasibility of forest-fire smoke detection using lidar. *International Journal of Wildland Fire*.

[5] Xian J., Xu W., Long C., Song Q., Yang S. (2020). Early forest-fire detection using scanning polarization lidar. *Applied Optics*.

[6] Fallows E. A., Cleary T. G., Miller J. H. (2009). Development of a multiple gas analyzer using cavity ringdown spectroscopy for use in advanced fire detection. *Applied Optics*.

[7] Wang J., Wang H. (2014). Tunable fiber laser based photoacoustic gas sensor for early fire detection. *Infrared Physics & Technology*.

[8] Chung Y. S., Le H. V. (1984). Detection of forest-fire smoke plumes by satellite imagery. *Atmospheric Environment*.

[9] Zhanqing Li Z., Khananian A., Fraser R. H., Cihlar J. (2001). Automatic detection of fire smoke using artificial neural networks and threshold approaches applied to AVHRR imagery. *IEEE Transactions on Geoscience and Remote Sensing*.

[10] Töreyin B. U., Cinbis R. G., Dedeoglu Y., Cetin A. E. (2007). Fire detection in infrared video using wavelet analysis. *Optical Engineering*.

[11] Muhammad K., Ahmad J., Mehmood I., Rho S., Baik S. W. (2018). Convolutional neural networks based fire detection in Surveillance videos. *IEEE Access*.

[12] Redmon J., Divvala S., Girshick R., Farhadi A. You only look once: Unified, real-time object detection[C].

[13] Park M., Ko B. C. (2020). Two-step real-time Night-time fire detection in an Urban environment using Static ELASTIC-YOLOv3 and Temporal fire-Tube. *Sensors*.

[14] Li P., Zhao W. (2020). Image fire detection algorithms based on convolutional neural networks. *Case Studies in Thermal Engineering*.

[15] Cai W., Wang C., Huang H., Wang T. A real-time smoke detection model based on YOLO-SMOKE algorithm[C].

[16] Liu Z., Lin Y., Cao Y. Swin transformer: hierarchical vision transformer using shifted windows[C].

[17] Xin F., Chuan L., Kai-Qun H. (2014). Infrared and visible image fusion based on deep Boltzmann model[J]. *Acta Physica Sinica*.

[18] Li X., Qin S.-Y. (2011). Efficient fusion for infrared and visible images based on compressive sensing principle. *IET Image Processing*.

[19] Redmon J., Farhadi A. (2018). Yolov3: An Incremental improvement[J]. https://arxiv.org/abs/1804.02767.

[20] Bochkovskiy A., Wang C. Y., Liao H. Y. M. (2020). Yolov4: Optimal Speed and Accuracy of Object detection[J]. https://arxiv.org/abs/2004.10934.

[21] Neubeck A., Van Gool L. Efficient non-maximum suppression[C].

[22] Girshick R. Fast R-CNN[C].

[23] Ramachandran P., Parmar N., Vaswani A., Bello I., Levskaya A., Shlens J. (2019). Stand-alone self-attention in vision models[J]. *Proc. Adv. Neural Inf. Process. Syst.*.

[24] Zhao H., Jia J., Koltun V. Exploring self-attention for image recognition[C].

[25] Srinivas A., Lin T. Y., Parmar N., Shlens J., Abbeel P., Vaswani A. Bottleneck transformers for visual recognition[C].

[26] Di Wu C. Z., Ji L., Ran R., Wu H., Xu Y. (2021). Forest fire recognition based on feature extraction from multi-view images. *Traitement du Signal*.

[27] Pinheiro P. O., Lin T.-Y., Collobert R., Dollár P. Learning to Refine Object segments[C].

[28] Li Z., Zhou F. (2017). FSSD: Feature Fusion Single Shot Multibox detector[J]. https://arxiv.org/abs/1712.00960.

